RETRACTED

# Evaluation of Hematological, Oxidative Stress, and Antioxidant Profile in Cattle Infected with Brucellosis in Southern Punjab, Pakistan

**DOI:** 10.1155/2022/7140909

**Published:** 2022-07-18

**Authors:** Riaz Hussain, Iahtasham Khan, Adil Jamal, Bahaeldeen Babiker Mohamed, Ahrar Khan

**Affiliations:** ^1^Department of Pathology, Faculty of Veterinary and Animal Sciences, The Islamia University of Bahawalpur, Bahawalpur 63100, Pakistan; ^2^Section of Epidemiology and Public Health, Department of Clinical Sciences, University of Veterinary and Animal Sciences, Lahore Sub-Campus Jhang 12-Km Chiniot Road, Jhang 35200, Pakistan; ^3^Sciences and Research, College of Nursing, Umm Al Qura University-715, Makkah, Saudi Arabia; ^4^Institute of Environment Natural Resources, The National Centre of Research, Khartoum, Sudan; ^5^Shandong Vocational Animal Science and Veterinary College, Weifang 261061, China; ^6^Faculty of Veterinary Science, University of Agriculture, Faisalabad, Pakistan

## Abstract

Brucellosis is a well-known and harmful zoonotic disease that poses a severe threat to public health and wild and dairy animals. Due to a lack of monitoring and awareness, disease incidence has increased. Therefore, this study was conducted for the first time to ascertain the status of seroprevalence of brucellosis, hematological, oxidative stress, and antioxidant enzymes in different breeds of cattle reared under tropical-desert conditions in Pakistan. This study comprised 570 cattle of different breeds. We recorded some epidemiological traits, including age and gender. The blood samples were obtained from all the cattle, screened with RBPT, and then confirmed by ELISA and PCR. The results recorded an overall 11.75%, 10.7%, and 9.64% prevalence of brucellosis based on RBPT, ELISA, and PCR. We obtained nonsignificant results in different age and sex groups of cattle. The results showed significantly (*P* ≤ 0.05) lower values of erythrocyte counts, hemoglobin quantity, hematocrit, lymphocytes, and monocytes in infected cases. The results showed that the total leukocyte and neutrophil cells significantly (*P* ≤ 0.05) increased. The lipid peroxidation parameters (MDA- and NO-scavenging activity of erythrocyte) increased significantly (*P* ≤ 0.05) in infected cattle, whereas significantly reduced antioxidant enzymes like SOD, RGSH, and CAT were. Similarly, significantly lower serum albumin levels and total serum proteins were recorded in infected cattle.

## 1. Introduction

Brucellosis is a zoonotic and contagious disease of wild and domestic animals and affects public health resulting in substantial economic losses. In livestock, it results in reduced productivity (20-25%), decreased milk production, abortion, and weak offspring and is a significant impediment to the trade [1, 2]. A high incidence of temporary and permanent infertility could result in the culling of animals. The disease has worldwide distribution and affects animals and humans in developed and developing countries [3, 4]. In developing countries, the disease burden is more profound due to inadequate public health measures, domestic animal health programs, and appropriate diagnostic facilities [5].

RETRACTED

Brucellosis caused by Brucella poses severe threats to public health worldwide [6]. However, its prevalence worldwide is highly prevalent in Mediterranean countries [7]. Brucella is an intracellular gram-negative bacterium and species-specific. The disease is caused by different species of Brucellae (nonmotile, anaerobic coccobacilli, and gram-negative), including two marine and six terrestrial species. Brucellosis is commonly transmitted via aborted fetuses, semen, uterine exudates, and fetal contents. In the male, brucellosis manifests permanent sterility, epididymitis, seminal vesiculitis, and orchitis [8]. In females, the disease causes death due to severe metritis, damage to fetal membranes, and retained placental contents. The exact mechanisms of pathogenesis of disease in animals are still under debate. Still, various studies have indicated that the causative agent enters the body via the digestive tract, mucosal layers, respiratory tract, and intact skin and spreads through the blood and lymphatic system to multiple tissues where it establishes the disease [9]. The infectious agent escapes from the phagocytizing and killing cells by inhibiting the phagosome-lysosome fusion and multiplication inside the macrophages [10].

In Pakistan, the prevalence of brucellosis increased over time, both in dairy animals and Equidae [11–13]. Brucella is commonly transmitted to humans by consuming raw milk and its products (milk cream, butter, and fresh cheese) or through contact with contaminated material. In Pakistan, work has been reported on the seroprevalence of brucellosis in cattle [14, 15], buffaloes [16], camels [17], dogs [18], equines [19–23], humans [13, 24, 25], and sheep and goats [26].

The maximum incidence of brucellosis in bovines ranged from 0.85% to 76% globally [27–30]. There are four provinces in Pakistan, i.e., Punjab, Balochistan, Sindh, and Khyber Pakhtunkhwa. In all livestock species in Pakistan, the seroprevalence of brucellosis is reported from zero to 76% [16, 30–37]. The highest (76%) seroprevalence of brucellosis was reported in goats, followed by bulk tank milk samples (42%) from Punjab, Pakistan [38]. During the preliminary assessment, it was reported that seroprevalence of brucellosis in different species was 0.00%, 0.23%, 3.41%, 26.19%, and 38.88% in sheep, goats, camels, cattle, and buffaloes, respectively [39]. Between KPK and Sindh, 11% and 21% of brucellosis prevalence have been reported [37, 38]. The overall prevalence of brucellosis in Baluchistan in small ruminants was 3.40% [40] and in large ruminants was 20% [25]. Many factors affect the prevalence of brucellosis, such as age, sex, species, different climatic conditions, geography, and diagnostic tests [3, 32, 41].

RETRACTED

It is an alarming situation that needs immediate attention. Most seroprevalence studies are based on RBPT and SAT; however, few studies are based on ELISA [1, 24, 25]. RBPT is based on the agglutination of serum antibodies with a stained whole cell preparation of killed *Brucella*. For confirmation of RBPT results, the serum agglutination test (SAT) or in more sophisticated equipped laboratories, ELISA may be used [42].

Monitoring oxidative stress, blood biochemistry, and defense system profile (antioxidant enzymes) are important tools to lower the adverse impacts of oxidative stress in animals. Studies have indicated that free radicals affect steroidogenesis, apoptosis, lipid peroxidation, and folliculogenesis leading to disorders in embryo preimplantation and infertility in animals [43–45]. Therefore, estimation of blood biochemistry, oxidative stress, and endogenous antioxidants are considered critical factors in initiating different molecular mechanisms during infectious diseases [46]. Scanty information is available in the published literature regarding the hematological, oxidative stress, and antioxidant profile in brucellosis-infected cattle. There is no information regarding brucellosis seroprevalence in cattle mainly kept in desert conditions, particularly in southern Punjab, Pakistan. Therefore, the present study has been planned to investigate the seroprevalence of brucellosis in food animals through serological and molecular-biological techniques.

## 2. Materials and Methods

### 2.1. Study Area and Animals

This study was conducted in three districts, including Lodhran, Bahawalpur, and Bahawalnagar of the Southern Punjab province. In Pakistan, about 52% of the agroecological area of Punjab province belongs to Southern Punjab and is inhabited by 32% of the total human population of the province. In southern Punjab, the desert area (Cholistan) lies between longitudes 69° 52′ to 75° 24′E and latitudes 27° 42′ 29°45′N and is comprised of three districts (Bahawalpur, Rahim Yar Khan, and Bahawalnagar).

The present study comprised 571 cattle of various breeds, including Cholistani (*n* = 163), Friesian (*n* = 148), Jersey (*n* = 123), and cross-bred (*n* = 137) cattle reared at three districts for the estimation of the burden of brucellosis.

RETRACTED

### 2.2. Blood Sampling and Screening of Brucellosis

We drew 5 mL of blood from the jugular vein of all the study animals separately. According to previous procedures, all the serum samples were subjected to RBPT and ELISA to detect brucellosis [23, 47]. We used an automated hematology analyzer for hematology. Take about 1 mL of collected blood to estimate various blood parameters like counting red blood cells, white blood cells, neutrophils, monocytes, lymphocytes, hemoglobin, and hematocrit. A total of 10 blood samples of each breed of healthy as control and brucellosis-positive cattle were used for hematological investigation.

### 2.3. Estimation of Oxidative Stress and Antioxidant Enzymes in Erythrocyte of Animals

Lipid peroxidation in the RBC hemolysate was identified as thiobarbituric acid reactive substance (TBARS) according to Grewal et al. [48]. The procedure depends on creating a color complex between thiobarbituric acid and the byproducts of lipid peroxidation (TBA). In a brief, 0.2 mL of RBC hemolysate was added to 1.3 mL of 0.2 M Tris-KCl buffer (pH 7.4), and the solution was then incubated at 37°C for 30 min before being heated in a boiling water bath for 10 min. After cooling, 3 mL of pyridine/n-butanol (3 : 1 *v*/*v*) and 1 mL of 1 N NaOH were added and mixed by continuous shaking. At 532 nm, the absorbance was measured using bidistilled water as a blank. 1,1,3,3-Tetramethoxypropane was utilized as a reference in this experiment. Lipid peroxidation in the RBC hemolysate was expressed as MDA nanomoles per grams of hemoglobin (nmol/gHb).

The activity of superoxide dismutase (SOD EC 1.15.1.1) was measured by the Misra and Fridovich method [49]. At 560 nm, the sample absorption was measured. Half of the rate of nitro blue tetrazolium (NBT) reduction is inhibited by one SOD activity unit. In a 1 cm cuvette, the NBT decrease rate is measured at 0.0165 absorbance units per minute. SOD activity was expressed as IU·mg^−1^ hemoglobin. Ransod (superoxide dismutase) control SD 126 from RANDOX Laboratories Ltd. was used to evaluate the method's accuracy.

By using a two-step colorimetric approach that was described by Asri-Rezaei and Dalir-Naghadeh [50], the activity of catalase was assessed. The samples were initially incubated with a known quantity of hydrogen peroxide since the rate of hydrogen peroxide dismutation to water and oxygen is proportional to the concentration of catalase. After a predetermined incubation time, the amount of hydrogen peroxide left was subsequently calculated by an oxidative coupling reaction involving 3,5-dicholo-2-hydroxybenzenesulfonic acid (DHBS) and 4-aminoantipyrene (4-AAP), which was accompanied by horseradish peroxide. The resulted quinoneimine dye was detected at 520 nm (Catalase Assay Kit, Oxford Biochemical Research, Inc., USA). The enzyme activities were measured in IU/mgHb.

RETRACTED

At physiological pH, nitric oxide produced from an aqueous sodium nitroprusside (SNP) solution reacts with oxygen to form nitrite ions, which can be measured and identified using the Griess Illosvoy reaction [51]. 10 mM SNP in 0.5 M phosphate buffer (pH 7.4) and different quantities (100-1000 g/mL) of MPE were included in the reaction mixture with final volume of 3 mL. Griess reagent (0.1 percent *α*-naphthyl-ethylenediamine in water and 1 percent sulphanilic acid in 5 percent H3PO4) was added following a 60-minute incubation period at 37°C. At 540 nm, spectrophotometric values were measured of the pink chromophore produced after the diazotization of nitrite ions with sulfanilamide and subsequent coupling with *α*-naphthyl-ethylenediamine. Ascorbic acid was used as a positive control. Nitric oxide scavenging ability (%) was calculated by using above percent inhibition (𝐼%) formula for DPPH assay.

The method of Asri-Rezaei and Dalir-Naghadeh [50], which is based on the production of a stable yellow hue when 2-nitrobenzoic acid is added to sulfhydryl compounds, was used to evaluate the activity of GSH-Px in the RBC hemolysate. The amounts of reduced product, thionitrobenzene, were measured by commercially available kits (Ransel test kit, Randox laboratories Ltd. GB) at 412 nm and express as IU/mgHb.

### 2.4. PCR-Based Confirmation of Brucella abortus

For confirmation of *Brucella abortus*, we extracted DNA. We performed PCR using specific primers (F = GAC GAA CGG AAT TTT TCC AAT CCC and R = TGC CGATCA CTT AAG GGC CTT CAT) as reported in a previous study [21]. Briefly, PCR reactions contained a total of 25 *μ*L reaction mixture having 1 *μ*L (dNTP), 1.2 *μ*L forward and reverse primers, and 1 *μ*L DNA template. The PCR amplification was carried out (35 cycles) with initial denaturation at 93°C for 5 min followed by denaturation at 90°C for 1 min, annealing at 58°C for 1 min, and elongation at 72°C for 1 min with final elongation at 72°C for 1 min.

### 2.5. Statistical Analysis

Data collected in this study were subjected to statistical software [52]. Data on some epidemiological traits, including age, species, and gender, were analyzed by chi-square. Data on blood, oxidative stress, and antioxidant parameters were subjected to by *t*-test.

## 3. Results

### 3.1. Brucellosis Prevalence in Cattle

The overall prevalence of brucellosis disease in dairy cattle has been shown in Table 1. The results showed an 11.75% disease prevalence based on RBPT, while the disease prevalence based on the ELISA test was 10.7%. Based on PCR techniques, the results recorded an overall 9.64% disease prevalence in dairy cattle. The results showed nonsignificantly occurring diseases in dairy cattle based on gender and age groups (Table 1).

RETRACTED

### 3.2. Hematological Parameters

The results of different hematological parameters of different dairy cattle breeds are presented in Table 2. The results revealed that the erythrocyte counts, hemoglobin quantity, hematocrit, lymphocytes, and monocytes decreased significantly (*P* ≤ 0.05) in all cattle breeds infected with brucellosis compared to healthy animals. The results showed that the total leukocyte and neutrophil cells significantly (*P* ≤ 0.05) increased in all cattle breeds infected with brucellosis compared to healthy animals.

### 3.3. Oxidative Stress Parameters and Antioxidant Enzymes

The results of different oxidative stress parameters and antioxidant enzymes in erythrocytes of brucellosis-infected and healthy cattle are presented in Table 3. The results on different oxidative stress parameters recorded in brucellosis-infected cattle indicated a substantial increase (*P* ≤ 0.05) in values of lipid peroxidation product (MDA) and nitric oxide scavenging activity in brucellosis-positive cattle as compared to healthy animals. The results on different antioxidant enzymes showed significantly (*P* ≤ 0.05) lower values of SOD, reduced glutathione, and CAT enzymes in erythrocytes of infected cattle as compared to healthy cattle. The results indicated significantly (*P* ≤ 0.05) lower serum albumin levels and total serum proteins in infected cattle compared to noninfected animals (Figure 1).

## 4. Discussion

Previously, 21.4% prevalence by RBPT of brucellosis and 3.56% by ELISA in equine animals kept in different districts of Punjab province, Pakistan, have been recorded [23]. In our study, no significant difference was recorded in the prevalence of disease based on different age groups of cattle. Previously, studies have recorded that the prevalence of brucellosis decreases due to advancement in the age of equines [23, 53, 54]. In contrast to our results, different earlier studies have found a significant association between the prevalence of brucellosis with age [8, 40, 55, 56]. The results showed a nonsignificant association of sex of animals regarding the presence of brucellosis in our study.

Similarly, no significant difference in the prevalence of brucellosis has also been recorded in animals [23]. An overall 12.7% prevalence of brucellosis in cattle kept in a periurban condition in Pakistan has also been reported [57]. At different livestock farms in Pakistan, up to 16.19% seroprevalence of brucellosis has been recorded in the cattle [3]. Compared to brucellosis in animals, a significantly increased prevalence of the disease has been recorded in females [14, 57, 58]. Variable prevalence of brucellosis includes 4.97% in goats and 5.6% in buffaloes using MRT, while 1.9% in buffaloes and 16.1% in goats with ELISA have been reported [47].

RETRACTED

Our study's hematological findings showed that the values of red blood cell count, hemoglobin quantity, and hematocrit significantly decreased in cattle of different breeds infected with brucellosis. Previously, scanty information was available regarding hematological changes in brucellosis-infected cattle [59]. Due to brucellosis in horses, lower erythrocyte sedimentation rate, basophils, and neutrophil counts have been reported [22]. Significantly reduced values of neutrophils, monocytes, and lymphocytes in brucellosis-infected cattle were seen. The increased neutrophil count in the present study could be related to oxidative stress leading to tissue damage. The lower values of lymphocytes and monocytes could be due to the poor immunological response of brucellosis-infected cattle. Few studies have reported that monocytosis mainly occurs due to damaged tissue debris in brucellosis animals' reproductive and urinary tract [60–62]. However, no report is available on the induction mechanisms of various hematological disorders in brucellosis-positive animals in published data. The changes in hematological parameters might be due to oxidative stress on bone marrow induction.

In the present study, the quantity of different antioxidant enzymes in erythrocytes of positive brucellosis cattle like RGSH, SOD, and CAT was significantly reduced (*P* ≤ 0.05). Previously, no information was available about the concentrations of different antioxidant enzymes in erythrocytes in brucellosis-positive animals. The lower concentrations of these antioxidant biomarkers in erythrocytes of brucellosis-positive cattle can be related to increased turnover of free radicals and depletion of antioxidants during disease prevention [63]. The lower values of various antioxidant enzymes in erythrocytes of brucellosis-positive cattle might be due to disorders in the physiological state and integrity of erythrocytic membranes due to low-grade inflammatory response resulting in inhibition of release of IL-1 and TNF-*α* [64].

Oxidative stress performs a vital role in the development of clinical disease and also leads to DNA damage, enzymic deactivation, lipid peroxidation, apoptosis, and cell necrosis [64–70]. With the declining body's antioxidant-based defense mechanism, oxidative stress concentration gets enhanced in brucellosis [71–73]. Before entrance in the macrophages, *Brucella* are opsonized inside the host with Brucella-specific immunoglobulin G (IgG), and the entrance into the macrophages is mainly because of phagocytosis initiated by Fc receptor. SOD, CAT, and glutathione peroxidase are vital antioxidant enzymes for the intracellular protection [65, 74]. The *Brucella* existence depends on the concentration of CAT and SOD in the *Brucella*. Of these, SOD performs a significant role in the pathophysiology of the *Brucella* [73].

RETRACTED

SOD catalyzes the transformation of superoxide radical to hydrogen peroxide [75] serving as the primary line of defense in response to oxidative stress [70], explaining why this enzyme showed high activity. SOD keeps the O_2_- levels under control in the cellular components and plays a crucial part in the death of phagocytosed bacteria intracellularly [72]. CAT is removed for the inhibition of OH- production that leads to formation of hydrogen peroxide in the cells. The hydrogen peroxide formed by SOD is degraded by the action of CAT, and it is able to cross the nuclear membrane and induce damage through enzymatic reactions [70, 75]. Thus, SOD and CAT are vital in the removal of nitrogen radicals and free oxygen produced by the Brucella, while glutathione peroxidase (GPx) handles the diminution hydroperoxides intracellularly [76, 77]. Glutathione peroxidase is another important antioxidant enzyme present intracellularly and is present within the cell in reduced form (GSH) as oxidants counter to endogenously formed peroxides. GPx catalyzes this reaction. To be able to effectively protect the cell, it is necessary that major part of glutathione has to be kept in reduced form [64, 78].

Brucella owns two SODs, SodA and SodC [73, 79], those directly cleanse radicals of superoxide. Superoxide cannot easily pass through with cellular membranes as being a charged molecule, and consequently, each SOD usually cleanses superoxide radical produced intracellularly in the bacterial components where they are present [80]. The lessening of *Brucella* in macrophages is also controlled by the acid-sensitive kind of the SodA transformed, thus are able to lower the oxygen readiness, and the reduced growth rate [81] may prevent endogenic superoxide concentration achieving an optimum level at which a cytoplasmic SOD cleanse in *Brucella* strains after setting up intracellularly in the host [65, 72].

The hydrogen peroxide generated during the process is deactivated by CAT. The CAT action is primarily limited to the Brucella's periplasm [82] and responsible to supply safety against H_2_O_2_ produced during immune reaction provoked against brucellosis. Control of CAT is necessary for the adjustment procedure of *Brucella* to endure and preserve under frightening circumstances. As CAT and Cu-Zn SOD are present at periplasmic location, thus are engaged in safeguarding the *Brucella* from peripheral oxidative complexes [82, 83]. In addition to this, a set of specific proteins are more sensitive to superoxide and activate signaling pathways and promote adaptation of elevated SODs or, alternatively, may initiate cellular death [84].

RETRACTED

Previous studies have investigated those lower concentrations of SOD, CAT, and RGSH in the erythrocytes of infected cattle, suggesting increased exposure of erythrocytes to oxidative stress and protecting effects of erythrocytes against oxidative damage [83]. Furthermore, a lower quantity of reduced glutathione might also be due to depletion of these enzymes during decomposition of lipid peroxidase and prevention of oxidative damage to membranes of red blood cells. The changes in host tissue and cells take place with increased concentration of oxidative stress parameters as a result of brucellosis [85]. The biomarkers of oxidative stress in brucellosis-positive cattle were significantly increased in the present study. The increased values of these biomarkers are suggestive of induction of oxidative stress and indicate that the increased process of oxidation in erythrocytes is responsible for the rapid generation of free radicals, ultimately leading to inefficient antioxidant capacity and breakdown of erythrocytes [72, 86]. It is further added as brucellosis renders low concentration of antioxidant enzymes; thus, oxidative enzymes (such as MDA, ceruloplasmin, NO, and Cu) increased [65]. Thus, increased oxidative stress leads to breakage of DNA, lipid peroxidation, and protein denaturation [64, 70, 87]; thus, total proteins and albumin were found to be lowered in brucellosis-infected cattle.

## 5. Conclusions

From the results, it was concluded that brucellosis is still prevailing in animals in Pakistan. Prevalence of cattle brucellosis was recorded to be 11.75%, 10.7%, and 9.64% based on RBPT, ELISA, and PCR, respectively. The hematological parameters studied including erythrocyte counts, hemoglobin quantity, hematocrit, lymphocytes, and monocytes significantly (*P* ≤ 0.05) reduced, whereas total leukocyte and neutrophils significantly increased in infected cases. The MDA and NO scavenging activity of erythrocyte increased significantly, while antioxidant enzymes (SOD, RGSH, and CAT) reduced significantly. Total serum proteins and albumin also lowered significantly in brucellosis-infected cattle.

RETRACTED

## Figures and Tables

**Figure 1:** Total proteins and albumin in brucellosis-negative and brucellosis-positive cattle. Note: the reading (mean ± SD) of total proteins and albumin is significantly (*P* ≤ 0.05) reduced in brucellosis-infected cows as compared to noninfected cows.

**Table 1:** RBPT-, ELISA-, and PCR-based prevalence of brucellosis in cattle kept at the Cholistan.

Species/sex/age	No. of animals	Positive		95% CI	Odd ratio/*P* value
		*N*	%		
RBPT test					
Sex					
Male	31	03	9.67	2.52-24.12	0.80 (reciprocal = 1.26)
Female	539	64	11.87	9.34-14.81	
Overall	570	67	11.75		
Age groups (years)					
3-4	167	13	7.78	4.40-12.63	Mantel-Haenszel chi-sq. *P* = 0.817
5-6	305	39	12.78	9.38-16.90	
>7	98	15	15.30	9.17-23.47	
ELISA					
Sex					
Male	31	02	6.45	1.10-19.72	0.56 (reciprocal = 1.78)
Female	539	59	10.94	8.51-13.80	
Overall	570	61	10.70		
Age groups (years)					
3-4	167	11	6.58	3.51-11.16	Mantel-Haenszel chi-sq. *P* = 0.611
5-6	305	36	11.80	8.53-15.80	
>7	98	14	14.28	8.37-22.29	
Polymerase chain reaction					
Sex					
Male	31	02	6.45	1.10-19.72	0.63 (reciprocal = 1.58)
Female	539	53	9.83	7.53-12.57	
Overall	570	55	9.64	7.42-12.28	
Age groups (years)					
3-4	167	09	5.38	2.66-9.66	Mantel-Haenszel chi-sq. *P* = 0.067
5-6	305	35	11.47	8.25-15.43	
>7	98	11	11.22	6.05-18.67	

**Table 2:** Blood profile (mean ± SD) of different breeds of cattle infected with brucellosis.

Cattle breed/parameters	Healthy	Infected	*P* value
Cholistani			
Erythrocyte counts (10^6^/*μ*L)	5.01 ± 0.15	3.69 ± 0.09	<0.01
Hemoglobin quantity (g/dL)	11.97 ± 1.12	8.19 ± 0.13	<0.01
Hematocrit (%)	34.50 ± 1.30	28.9 ± 2.3	<0.01
Leukocyte counts (10^3^/*μ*L)	9.11 ± 0.89	13.83 ± 0.71	<0.01
Neutrophil (%)	19.70 ± 1.90	25.9 ± 1.7	<0.01
Lymphocyte (%)	49.80 ± 3.70	31.5 ± 1.83	<0.01
Monocyte (%)	6.33 ± 0.15	4.01 ± 0.07	<0.01
Jersey			
Erythrocyte counts (10^6^/*μ*L)	5.17 ± 0.13	3.81 ± 0.05	<0.01
Hemoglobin quantity (g/dL)	12.09 ± 0.93	7.97 ± 0.41	<0.01
Hematocrit (%)	36.77 ± 2.05	28.24 ± 2.75	<0.01
Leukocyte counts (10^3^/*μ*L)	10.07 ± 1.03	16.19 ± 1.07	<0.01
Neutrophil (%)	21.23 ± 2.19	31.29 ± 2.13	<0.01
Lymphocyte (%)	53.40 ± 2.40	37.3 ± 2.3	<0.01
Monocyte (%)	5.59 ± 0.31	3.97 ± 0.23	<0.01
Cross-bred			
Erythrocyte counts (10^6^/*μ*L)	5.33 ± 0.19	3.92 ± 0.11	<0.01
Hemoglobin quantity (g/dL)	13.01 ± 1.03	8.55 ± 0.33	<0.01
Hematocrit (%)	37.13 ± 3.11	26.39 ± 3.03	<0.01
Leukocyte counts (10^3^/*μ*L)	12.13 ± 0.91	17.03 ± 0.03	<0.01
Neutrophil (%)	23.49 ± 3.33	39.01 ± 4.51	<0.01
Lymphocyte (%)	46.91 ± 3.70	34.90 ± 3.25	<0.01
Monocyte (%)	5.73 ± 0.19	3.99 ± 0.03	<0.01
Friesian			
Erythrocyte counts (10^6^/*μ*L)	4.99 ± 0.07	3.59 ± 0.11	<0.01
Hemoglobin quantity (g/dL)	13.01 ± 0.03	9.05 ± 0.29	<0.01
Hematocrit (%)	35.03 ± 1.19	27.03 ± 1.07	<0.01
Leukocyte counts (10^3^/*μ*L)	11.07 ± 0.07	17.01 ± 0.87	<0.01
Neutrophil (%)	24.11 ± 1.15	39.01 ± 1.01	<0.01
Lymphocyte (%)	55.11 ± 3.13	39.1 ± 3.02	<0.01
Monocyte (%)	4.93 ± 0.57	3.63 ± 0.29	<0.01

RETRACTED

**Table 3:** Oxidative stress and antioxidant parameters (mean ± SD) of brucellosis-positive and brucellosis-negative cattle.

Parameters	Noninfected	Infected	*P* value
Oxidative stress biomarkers			
MDA (nmol/gHb)	1.54 ± 0.11	2.030 ± 0.08	<0.01
NO scavenging activity (%)	21.36 ± 0.40	28.71 ± 3.50	<0.001
Antioxidant biomarkers			
SOD (IU/mgHb)	142.40 ± 9.80	121.50 ± 2.10	<0.01
RGSH (IU/mgHb)	171.40 ± 7.10	151.70 ± 2.60	<0.001
CAT (IU/mgHb)	131.30 ± 6.70	105.40 ± 2.20	<0.01

## Data Availability

All the data related to the study is mentioned in the manuscript.

## Abbreviations

ALB: Albumin
CAT: Catalase
ELISA: Enzyme-linked immunosorbent assay
IgG: Immunoglobulin G
IL-1: Interleukin-1
MDA: Malondialdehyde
MRT: Milk ring test
NO: Nitric oxide
PCR: Polymerase chain reaction
RBPT: Rose Bengal precipitation test
RGSH: Reduced glutathione
SOD: Superoxide dismutase
TNF-*α*: Tissue necrosis factor alpha.
